# Segmentation Algorithm-Based Safety Analysis of Cardiac Computed Tomography Angiography to Evaluate Doctor-Nurse-Patient Integrated Nursing Management for Cardiac Interventional Surgery

**DOI:** 10.1155/2022/2148566

**Published:** 2022-05-04

**Authors:** Aiqiong Zhang, Qiuxiang Chen

**Affiliations:** ^1^Intervention Section, South Hospital of Chenzhou First People's Hospital, Chenzhou, 423000 Hunan, China; ^2^Operation Room, South Hospital of Chenzhou First People's Hospital, Chenzhou, 423000 Hunan, China

## Abstract

To deeply analyze the influences of doctor-nurse-patient integrated nursing management on cardiac interventional surgery, 120 patients with coronary heart disease undergoing cardiac interventional therapy were selected as the subjects and randomly divided into two groups, 60 cases in each group. The experimental group used the doctor-nurse-patient integrated nursing, while the control group adopted the routine nursing. The Hessian matrix enhanced filter segmentation algorithm was used to process the cardiac computed tomography angiography (CTA) images of patients to assess the algorithm performance and the safety of nursing methods. The results showed that the Jaccard, Dice, sensitivity, and specificity of cardiac CTA images of patients with coronary heart disease processed by Hessian matrix enhanced filter segmentation algorithm were 0.86, 0.93, 0.94, and 0.95, respectively; the disease self-management ability score and quality of life score of patients in the experimental group after nursing intervention were significantly better than those before nursing intervention, with significant differences (*P* < 0.05). The number of cases with adverse vascular events in the experimental group was 3 cases, which was obviously lower than that in the control group (15 cases). The diagnostic accuracy of the two groups of patients after segmentation algorithm processing was 0.87 and 0.88, respectively, which was apparently superior than the diagnostic accuracy of conventional CTA (0.58 and 0.61). In summary, cardiac CTA evaluation of doctor-nurse-patient integrated nursing management cardiac interventional surgery based on segmentation algorithm had good safety and was worthy of further promotion in clinical cardiac interventional surgery.

## 1. Introduction

Atherosclerotic lesion of coronary artery is a kind of heart disease caused by coronary artery organic (atherosclerosis or dynamic vasospasm) stenosis or vascular obstruction, leading to myocardial ischemia and hypoxia or myocardial necrosis, known as coronary atherosclerotic heart disease [1]. It, together with functional changes (spasm), inflammation, embolism, and congenital malformations of the coronary arteries, is collectively referred to as coronary heart disease or ischemic heart disease [2]. Atherosclerotic lesions of the coronary arteries are classified as occult, angina, myocardial infarction, heart failure and arrhythmia, and sudden death. The most common of these is the angina type, and the most severe are two types: myocardial infarction and sudden death [3, 4].

At present, the treatment methods for coronary heart disease include drug therapy and surgical treatment. In the rescue process of patients with acute myocardial infarction, percutaneous coronary intervention (PCI) is a common treatment method. This method is to intervene the special stent or balloon in the blocked vessel of the patient by the doctor, and use the stent or dilated balloon to support the plaque that has been detached and stabilize it again, so as to achieve the purpose of treatment [5]. Studies pointed out that current PCI is divided into primary PCI (PCI performed directly without thrombolytic therapy), rescue PCI, and PCI in recanalization of thrombolytic therapy [6]. Among them, primary PCI is indicated for patients within 12 hours of symptom onset and with persistent new left bundle branch block or evidence of myocardial ischemia (still with chest pain and ECG changes) within 12 to 48 hours; rescue PCI is indicated for patients with significant chest pain after thrombolytic therapy and no significant recovery of ECG parameters; PCI for patients with recanalization of thrombolytic therapy is indicated for emergency angiography after successful thrombolysis, and infarct-related artery revascularization therapy can be performed when necessary to relieve myocardial ischemia caused by severe residual stenosis [7, 8]. However, the risk of thrombosis and in-stent restenosis occurs after PCI. Timely and effective postoperative care and cardiac rehabilitation training play an important role in ensuring the effect of PCI treatment and improving the prognosis of patients. Routine nursing is usually followed by medical care, with weak individual pertinence, which cannot meet the nursing needs of all patients, while doctor-nurse-patient integrated nursing is an integrated nursing model combining doctor-nurse-patient. It can effectively allocate medical care resources and improve the quality of clinical nursing and nursing satisfaction and has been more and more widely used in clinical practice [9, 10].

Coronary computed tomography angiography (CTA) images are angiographic images produced by MSCT, and the patient's heart region is scanned by MSCT to obtain hundreds of images with 512∗512 resolution at one time. These images are characterized by high resolution and low noise. By virtue of the contrast agent component in the blood, the vascular and ventricular regions in the congested state have higher brightness than other parts [11]. However, the CTA images obtained by MSCT are only the information of the axial plane of the patient's heart site, and clinicians need to observe from the continuous two-dimensional images of a certain tomography and judge them according to their own experience, and the diagnostic results have great subjective experience, so the upgraded image identification and processing means are urgent problems to be solved at present [12, 13].

Convolutional neural network (CNN) algorithm based on deep learning, clustering, random forest classifier, and Hessian matrix algorithm are often used to solve various lesion segmentation problems in the currently reported medical image region segmentation methods. Studies indicated that the eigenvalues of the Hessian matrix can be used to identify tubular targets in images, and this algorithm can be regarded as a filter for vascular enhancement, with Gaussian multiscale fusion, to achieve effective enhancement of vascular images of different sizes [14, 15]. At present, there is no relevant study on the processing of cardiac CTA images by Hessian matrix segmentation algorithm for patients with coronary heart disease before and after integrated nursing and cardiac interventional therapy. Therefore, this study hopes to design a Hessian matrix filtering enhanced segmentation algorithm for the vascular image characteristics of patients with coronary heart disease under CTA images and use it in the CTA image diagnosis of patients with clinical coronary heart disease. By evaluating the algorithm performance and comparing the diagnostic accuracy, the application potential of this algorithm is comprehensively assessed. In addition, this algorithm will be adopted to evaluate the effect and safety of doctor-nurse-patient integrated nursing on cardiac treatment of coronary heart disease.

To sum up, a total of 120 patients with coronary heart disease and performed with PCI treatment were included as the research objects. They all participated in segmentation model-based cardiac CTA examination. Besides, all the patients were divided into experimental group (60 cases receiving doctor-nurse-patient integrated nursing) and control group (60 cases receiving conventional nursing) according to different nursing methods to deeply assess the application effects of doctor-nurse-patient integrated nursing management in cardiac interventional surgery, which was aimed at providing help for the clinical diagnosis and treatment of coronary heart disease.

## 2. Materials and Methods

### 2.1. Study Subjects

A total of 120 patients with coronary heart disease in hospital from March 2019 to March 2021 were selected as the study subjects, and all patients were examined by cardiac CTA. The age range of patients was 43-79 years; the mean age was 61.35 ± 6.42 years. There were 74 males and 46 females. The disease course of patients was between 1 and 14 years, with a mean disease course of 5.46 ± 2.42 years. This study had been approved by the ethics committee of hospital, and all subjects signed the informed consent form.

Inclusion criteria are as follows: (1) patients who meet the relevant WHO diagnostic criteria for coronary heart disease, namely, coronary angiography has more than one coronary artery diameter stenosis ≥ 50% and (2) patients with stable postoperative condition and cooperate with the treatment. Exclusion criteria are as follows: (1) patients with contraindications to interventional surgery; (2) patients combined with other mental diseases, cognitive impairment, or communication disorders; and (3) patients combined with other severe chronic diseases.

### 2.2. Grouping and Nursing Method Selection

The patients with coronary heart disease treated with PCI were randomly divided into two groups, with 60 patients in each group, one of which was treated with routine nursing and the other with doctor-nurse-patient integrated nursing. Among them, routine nursing includes guiding the patient's postoperative medication, diet, exercise, and other conditions and telling them to return regularly. The integrated nursing of doctor-nurse-patient means that specialists are responsible for popularizing the common problems of coronary heart disease, advantages, and limitations of interventional surgery and providing some medical suggestions for patients. Responsible nurses remind patients to take medicine according to the doctor's advice, regularly monitor various indicators of patients, conduct emotional counseling for patients, provide patients with diet and rehabilitation exercise guidance, establish a timely communication mechanism between doctors, nurses, and patients, and do a good job in return visit after patients are discharged.

### 2.3. Establishment of Cardiac CTA Segmentation Model Based on Hessian Matrix Enhanced Filtering Segmentation Algorithm

The current study confirmed that the Hessian matrix enhanced filtering can accurately identify the tubular structure in the image and can also show a significant enhancement effect under multiscale conditions [16]. Therefore, in this study, it is hoped to use a single-scale Hessian matrix enhanced filtering algorithm to effectively distinguish the vascular structure and background in CTA images. Then, the center of the ascending aorta was used as the seed point to segment the coronary artery and ascending aorta using regional growth, followed by the cavity filling algorithm to repair the problem of thick vessel internal cavities caused by single-scale Hessian matrix enhanced filtering.  Figure 1 is a schematic diagram of the cardiac CTA segmentation process for the Hessian matrix enhanced filtering segmentation algorithm.

Taylor series expansion is used in the analysis of the local features of the CTA three-dimensional image. The image is set as the point *B* in the *M* field, and Taylor series expansion is shown in Equation (1), and the three-dimensional Hessian matrix expression is shown in Equation (2).

(1) $$\begin{array}{c} M\left(B+\Delta B\right)\approx M\left(B\right)+\Delta B^{T}\nabla M\left(B\right)+\Delta B^{T}H\left(B\right)\Delta B, \end{array}$$

(2) $$\begin{array}{c} H\left(B\right)=\left[\begin{array}{ccc} I_{xx}\left(B\right) & I_{xy}\left(B\right) & I_{xz}\left(B\right)\\ I_{yx}\left(B\right) & I_{yy}\left(B\right) & I_{yz}\left(B\right)\\ I_{zx}\left(B\right) & I_{zy}\left(B\right) & I_{zz}\left(B\right) \end{array}\right]. \end{array}$$

In Equation (1), the coordinate of point *B* is expressed as (*x*, *y*, *z*). In the two-dimensional image *B* = (*x*, *y*), ∇*M*(*B*) represents the gradient of the image at point *A*, and *H* (*B*) represents the Hessian third-order symmetric matrix of point *B*. In Equation (2), *I*_*xx*_(*B*), *I*_*xy*_(*B*), *I*_*xz*_(*B*), *I*_*yx*_(*B*), *I*_*yy*_(*B*), *I*_*yz*_(*B*), *I*_*zx*_(*B*), *I*_*zy*_(*B*), and *I*_*zz*_(*B*) represent the second-order partial derivatives of the three-dimensional image at point *B*, respectively. The three eigenvalues of the Hessian third-order symmetric matrix *H* (*B*) are denoted as *λ*_1_, *λ*_2_, and *λ*_3_. The corresponding eigenvectors are expressed as *v*_1_, *v*_2_, and *v*_3_. The absolute value of the eigenvalues represents the intensity. The eigenvector corresponding to the eigenvalue with the largest absolute value corresponds to the maximum curvature direction of the three-dimensional surface at this point. The eigenvector corresponding to the eigenvalue with the smallest absolute value corresponds to the tangent direction of the three-dimensional surface at this point and corresponds to the actual direction of the blood vessel. Usually, the absolute values and eigenvalues in two-dimensional and three-dimensional images satisfy Equations (3) and (4).

(3) $$\begin{array}{c} \left|\lambda_{1}\right|\leq \left|\lambda_{2}\right|, \end{array}$$

(4) $$\begin{array}{c} \left|\lambda_{1}\right|\leq \left|\lambda_{2}\right|\leq \left|\lambda_{3}\right|. \end{array}$$

The vascular structure in the ideal state is tubular. The vascular structure is analyzed by the eigenvalues of the Hessian matrix, and the corresponding eigenvalues of the vascular structure can be expressed as Equation (5). On this basis, the Hessian matrix eigenvalues are used to construct a filter to enhance the vascular structure. The similarity function of blood vessels in three-dimensional images can be expressed as Equation (6).

(5) $$\begin{array}{c} \left\{\begin{array}{c} \left|\lambda_{1}\right|\approx 0,\\ \left|\lambda_{1}\right|\ll \left|\lambda_{2}\right|,\\ \left|\lambda_{2}\right|\approx \left|\lambda_{3}\right|, \end{array}\right. \end{array}$$

(6) $$\begin{array}{c} v\left(\lambda \right)=\left\{\begin{array}{cc} 0 & \text{if}\lambda_{2}>0\text{or}\lambda_{3}>0,\\ \left(1-\exp\left(-\frac{S_{B}^{2}}{2\alpha^{2}}\right)\right)\exp\left(-\frac{S_{C}^{2}}{2\beta^{2}}\right)\left(1-\exp\left(-\frac{W}{2\varepsilon^{2}}\right)\right) & \text{else}. \end{array}\right. \end{array}$$

In Equation (6), *S*_*B*_ and *S*_*C*_ represent the parameters corresponding to the ellipsoid model, respectively, which can reflect the difference between tubular structure, patchy structure, and disc structure, and *S*_*B*_ means the relationship between the semimajor axis of the ellipsoid and the cross section perpendicular to the vascular direction. *α*, *β*, *ε*, and *W* are the vascular parameters, and the corresponding expressions of *S*_*B*_, *S*_*C*_, and *W* are found in Equations (7)–(9).

(7) $$\begin{array}{c} S_{B}=\frac{Q/\pi }{L^{2}}=\frac{\left|\lambda_{2}\right|}{\left|\lambda_{3}\right|}, \end{array}$$

(8) $$\begin{array}{c} S_{C}=\frac{V/\left(4\pi /3\right)}{{\left(Q/\pi \right)}^{3/2}}=\frac{\left|\lambda_{1}\right|}{\sqrt{\left|\lambda_{2}\lambda_{3}\right|}}, \end{array}$$

(9) $$\begin{array}{c} W=\sqrt{{\lambda_{1}}^{2}+{\lambda_{2}}^{2}+{\lambda_{3}}^{2}}. \end{array}$$

*Q* indicates the maximum cross-section perpendicular to the direction of the vessel, *L* indicates the length of the semimajor axis, and *V* denotes the volume of the ellipse. Due to the different vascular scale, the response effect of the Hessian matrix filter to enhance the vascular structure is greatly reduced. Therefore, the CNN technology is introduced. The Gaussian function (Equation (10)) is used to convolution the target image, and the second derivative is calculated on the basis of the image. Equation (11) is used to solve it, and the vascular similarity function under this condition is shown in Equation (12).

(10) $$\begin{array}{c} H\left(B,\omega \right)=\exp\left(-\frac{B^{2}}{2\omega^{2}}\right), \end{array}$$

(11) $$\begin{array}{c} I_{xx}=I\left(B\right)*\frac{\partial^{2}H\left(B,\omega \right)}{\partial x^{2}}, \end{array}$$

(12) $$\begin{array}{c} v=\max\omega_{\min}\leq \omega \leq \omega_{\max}v\left(\omega ,\lambda \right). \end{array}$$

*ω* denotes the size of the Gaussian kernel and the scale of this filter. The maximum response value of vascular structure at different scales can be tested using different *ω*, so as to make the filtering enhancement effect of vessels at different scales more obvious.

Afterwards, the enhanced images of each layer of blood vessels are subjected to Hoff transform to obtain the seed points of the left and right coronary arteries, and then, the image hierarchy is superimposed to obtain the two-dimensional images generated by three-dimensional region growth. In addition, two-dimensional cavity filling algorithm is also used in this study to improve the internal cavity problem of thick blood vessels. The algorithm distinguishes the binary value of the front attraction and the background point of pixels in the CTA image, while some background points at the location of the cavity are surrounded by the front attraction. According to the characteristics, the replacement rule of the background point to the front attraction is set. If the number of front attractions in a neighborhood pixel is greater than the number of background points, the background points can be replaced into front attractions. For example, in a 3∗3 field, any background point has eight adjacent pixels, and as long as the number of front attractions in the adjacent pixels that meet the point is not less than 4, the point can be replaced into a front attraction (Figure 2).

### 2.4. Segmentation Quality Evaluation of Cardiac CTA Images Based on Hessian Matrix Enhanced Filtering Segmentation Algorithm

CNN algorithm [17] and V-net network (V-net) algorithm [18] were introduced to be compared with the proposed Hessian matrix enhanced filtering segmentation algorithm. In this study, Jaccard index, Dice similarity coefficient, sensitivity, and specificity were used to express the effect of coronary artery segmentation, and the range of the two values was between 0 and 1, and the higher the value, the higher the segmentation accuracy.

(13) $$\begin{array}{c} \text{Jaccard}=\frac{\left|A\cap B\right|}{\left|A\right|\cup \left|B\right|}, \end{array}$$

(14) $$\begin{array}{c} \text{Dice}=\frac{2\left|A\cap B\right|}{\left|A\right|+\left|B\right|}, \end{array}$$

(15) $$\begin{array}{c} \text{Sensitivity}=\frac{\text{TP}}{\text{TP}+\text{FN}}, \end{array}$$

(16) $$\begin{array}{c} \text{Specificity}=\frac{\text{TN}}{\text{TN}+\text{FP}}. \end{array}$$

In Equations (13) and (14), *A* is the true result and *B* is the predicted segmentation result. TP represents that the position that is originally a vascular point is correctly segmented into the pixel number of a vascular point, FP represents that the position that is originally a vascular point is incorrectly segmented into the pixel number of a nonvascular point, TN expresses that the position that is originally a nonvascular point is correctly segmented into the pixel number of a nonvascular point, and FN expresses that the position that is originally a nonvascular point is incorrectly segmented into the pixel number of a vascular point.

### 2.5. Diagnostic Effect Analysis of Cardiac CTA Image Based on Hessian Matrix Enhanced Filtering Segmentation Algorithm

The pathological diagnostic results were viewed as gold standard. The accurate results of the diagnosis by cardiac CTA images for myocardial infarction patients before and after the processing by Hessian matrix enhanced filtering segmentation algorithm were summarized to calculate the diagnostic accuracy.

### 2.6. Statistical Methods

The test data were processed by the SPSS 19.0 statistical software. The measurement data were expressed as mean ± standard deviation ($\overset{¯}{x}\pm s$). The comparison of mean between groups was performed by *t* test. The enumeration data were expressed as percentage (%). The *χ*^2^ test was used. The differences were statistically significant when *P* < 0.05.

## 3. Results

### 3.1. Basic Information of Patients

Figure 3 shows the comparison diagram of the basic situation of the two groups of patients. There were 36 male and 24 female patients in the experimental group and 38 male and 22 female patients in the control group, and there was no significant difference in the gender ratio between the two groups (*P* > 0.05). The mean age of the patients in the experimental group was 59.86 ± 7.38 years, and the mean disease duration was 5.18 ± 2.53 years; the mean age of the patients in the control group was 61.86 ± 6.57 years, and the mean disease duration was 5.65 ± 2.37 years. There was no significant difference in the mean age and mean disease duration between the two groups (*P* > 0.05).

### 3.2. Processing Results of Cardiac CTA Images Based on Hessian Matrix Enhanced Filtering Segmentation Algorithm

Figure 4 suggests the cardiac CTA image maps of the two groups of patients before and after processing by the Hessian matrix enhanced filtering segmentation algorithm.

### 3.3. Image Quality Evaluation of Cardiac CTA Processed by Different Algorithms

Figure 5 is the image quality comparison of cardiac CTA processed by different algorithms. Relative to the traditional CNN algorithm (0.74, 0.79, 0.72, and 0.75) and V-net algorithm (0.79, 0.84, 0.79, and 0.81), the Jaccard, Dice, sensitivity, and specificity (0.86, 0.93, 0.94, and 0.95) of cardiac CTA images of patients with coronary heart disease processed based on Hessian matrix enhanced filtering segmentation algorithm were significantly improved, and the differences were statistically significant (*P* < 0.05).

### 3.4. Comparison of Disease Self-Management Ability and Quality of Life before and after Nursing Intervention between the Two Groups

Figure 6 reveals the comparison diagram of disease self-management ability before and after intervention between the two groups, and Figure 7 reveals the comparison diagram of quality of life before and after nursing intervention between the two groups. In the evaluation of disease self-management ability before and after routine nursing intervention, the scores of daily life, disease medicine, and emotional management in the control group did not show significant changes, while the scores of those and the total score of disease self-management ability in the experimental group showed significant improvement before and after the integrated doctor-nurse-patient nursing intervention (Figure 5), and the differences were statistically significant (*P* < 0.05). There was no significant difference between the quality of life scores of the experimental group and the control group before the nursing intervention (*P* > 0.05), while the physical function, physical function, physical pain, vitality, social function, emotional function, mental health, and general health status scores of the quality of life assessment indicators of the experimental group and the control group showed significant differences after the nursing intervention (*P* < 0.05).

### 3.5. Incidence of Adverse Reactions in the Two Groups

Figure 8 suggests the occurrence of adverse vascular events in the two groups. In the experimental group, there were a total of 2 cases of stent stenosis, 1 case of recurrent angina pectoris, and 0 case of nonfatal myocardial infarction, and a total of 3 patients had adverse vascular reactions, while in the control group, there were a total of 5 cases of stent stenosis, 6 cases of recurrent angina pectoris, and 4 cases of nonfatal myocardial infarction, and a total of 15 patients had adverse vascular events. The comparison showed that the incidence rate of various types of adverse vascular events in the experimental group was significantly lower than that in the control group, and the difference had statistical significance (*P* < 0.05).

### 3.6. Diagnostic Accuracy of CTA Images before and after Processing by Segmentation Algorithm in the Two Groups

Figure 9 suggests the diagnostic accuracy of CTA images before and after processing by segmentation algorithm in the two groups. The disease diagnostic accuracy of the experimental group and the control group before processing by the Hessian matrix enhanced filtering segmentation algorithm was 0.58 and 0.61, respectively, while the disease diagnostic accuracy of the experimental group and the control group after processing by the segmentation algorithm was 0.87 and 0.88, respectively. It was found that the diagnostic accuracy of the patients with coronary heart disease after processing by the segmentation algorithm was significantly superior than that before processing, and the difference was statistically meaning (*P* < 0.05).

## 4. Discussion

Coronary heart disease, as one of the most prevalent cardiac diseases in China, is currently treated with three main treatment methods, which are drug therapy, coronary artery bypass grafting, and interventional therapy, of which interventional therapy refers to the treatment method in which transcatheter techniques dredge the stenotic or even occluded coronary arteries, thereby improving myocardial blood perfusion. This technology has the most significant advantages and rapid development and is one of the most used treatments for modern coronary heart disease treatment [19]. With the advancement of modern medical equipment and technology, especially the application of drug-eluting stents, the success rate of interventional therapy for coronary heart disease can reach more than 95%. In addition, various complications concerned by many patients can also be controlled within 5% [20]. However, because each surgery has certain risks, comprehensive and effective preoperative disease evaluation and prognosis detection are very critical for clinical treatment. At present, ECG, myocardial markers, coronary angiography, and other examinations are often adopted to diagnose coronary heart disease in clinical practice [21].

In this study, a Hessian matrix enhanced filtering segmentation algorithm was designed for CTA images of patients with coronary heart disease, which is used in the clinical diagnosis of patients with coronary heart disease who have undergone cardiac interventional surgery. By evaluating the algorithm performance and comparing the diagnostic accuracy, the application potential of this algorithm was comprehensively evaluated, and this algorithm was utilized to evaluate the effect and safety of different nursing methods on the cardiac treatment of coronary heart disease. The results revealed that Jaccard, Dice, sensitivity, and specificity (0.86, 0.93, 0.94, and 0.95) of cardiac CTA images of patients with coronary heart disease based on Hessian matrix enhanced filtering segmentation algorithm were all obviously enhanced compared with those based on traditional CNN algorithm (0.74, 0.79, 0.72, and 0.75) and on V-net algorithm (0.79, 0.84, 0.79, and 0.81). The differences were remarkable, which indicated statistical meaning (*P* < 0.05). It indicates that the Hessian matrix enhanced filtering segmentation algorithm designed in this study is further improved and upgraded on the basis of the traditional segmentation algorithm, significantly improves the segmentation accuracy of cardiac CTA images in patients with coronary heart disease under the computer program. Moreover, the algorithm further realizes the accurate identification and segmentation of vascular imaging in patients with coronary heart disease and contributes to the clinical diagnosis of the disease [22].

The patients in the experimental group showed significant improvement in daily life, disease medicine, emotional management score, total score of disease self-management ability, and quality of life score before and after doctor-nurse-patient integrated nursing intervention, and the differences were statistically significant (*P* < 0.05). The patients in the control group showed significant changes in disease self-management ability score and quality of life score before and after routine nursing intervention, thus indicating that in contrast to routine nursing, the doctor-nurse-patient integrated nursing model can improve the disease self-management ability and quality of life of patients with coronary heart disease treated with interventional surgery. In this study, by comparing the one-year adverse vascular events between routine nursing and integrated nursing, it was found that the prognosis of patients in the experimental group showed 2 cases of stent stenosis, 1 case of angina pectoris recurrence, and 0 case of nonfatal myocardial infarction, and a total of 3 patients had adverse vascular reactions, while the prognosis of patients in the control group showed 5 cases of stent stenosis, 6 cases of angina pectoris recurrence, and 4 cases of nonfatal myocardial infarction, and a total of 15 patients had adverse vascular events. The comparison meant that the incidence rate of various types of adverse vascular events in the experimental group was significantly inferior than that in the control group, and the difference had statistical significance (*P* < 0.05). It reveals that compared with routine care, integrated care will significantly reduce the probability of adverse vascular events in the prognosis of patients with coronary heart disease undergoing interventional surgery and improve the safety of the prognosis of patients, which is consistent with the results of Watts et al. [23]. In this study, the diagnostic accuracy of the two groups of patients before and after segmentation algorithm processing was compared. The results found that the diagnostic accuracy of patients with coronary heart disease after segmentation algorithm processing was significantly higher than that before processing (*P* < 0.05). It indicates that the Hessian matrix enhanced filtering segmentation algorithm designed in this study can significantly improve the clinical diagnostic accuracy of the disease when processing CTA images of patients with coronary heart disease, which is worthy of promotion.

## 5. Conclusion

A Hessian matrix filtering enhanced segmentation algorithm that could be used for CTA images of patients with coronary heart disease was designed and applied in the clinical nursing of patients with coronary heart disease and performed with cardiac interventional surgery. The final results demonstrated that Hessian matrix filtering enhanced segmentation algorithm could obviously improve the segmentation effect and diagnostic accuracy of CTA images of patients with coronary heart disease. Doctor-nurse-patient integrated nursing could effectively enhance patients' self-management ability and quality of life and reduce the incidence of adverse prognostic vascular events. The shortcomings of this study are that the number of included patients with coronary heart disease is small, the corresponding results of different nursing of patients with different types of coronary heart disease after interventional surgery are not compared and analyzed, and it is hoped that more relevant patient data will be collected in the future, and the above problems will be further studied. In conclusion, this study confirms the CTA image processing ability of the Hessian matrix filtering enhanced segmentation algorithm and the clinical value of doctor-nurse-patient integrated nursing intervention, which provides new ideas for the clinical diagnosis and treatment of coronary heart disease.

## Figures and Tables

**Figure 1:** CTA coronary artery segmentation flow chart.

**Figure 2:** 3∗3 neighborhood diagram.

**Figure 3:** Basic information of patients in the two groups. (a) The gender distribution map of patients in the two groups; (b) the mean age and mean disease course distribution map of patients in the two groups.

**Figure 4:** Cardiac CTA image of two groups of patients before and after processing by Hessian matrix enhanced filtering segmentation algorithm. (a, b) The CTA images of the experimental group patients before and after processing by the Hessian matrix enhanced filtering segmentation algorithm, respectively; (c, d) the CTA images of the control group patients before and after processing by the Hessian matrix enhanced filtering segmentation algorithm, respectively.

**Figure 5:** MRI image diagram processed by different algorithms. ∗ indicates that there is a statistically significant difference (*P* < 0.05) in the image quality indicators compared with conventional CNN algorithm and V-net algorithm.

**Figure 6:** Comparison of disease self-management ability before and after nursing intervention between the two groups. (a) Comparison of daily life management scores before and after nursing intervention between the two groups; (b) comparison of disease medical management scores before and after nursing intervention between the two groups; (c) comparison of emotional management scores before and after nursing intervention between the two groups; (d) comparison of total self-management ability scores before and after nursing intervention between the two groups; ∗ indicates significant difference in contrast to before nursing intervention (*P* < 0.05).

**Figure 7:** Comparison of quality of life before and after nursing intervention between the two groups. (a) Comparison of quality of life scores before nursing intervention between the two groups; (b) A–H refer to physiological function, physiological role, body pain, vitality, social function, affective role, mental health, and general health status, respectively. ∗ indicates significant difference in quality of life scores versus the control group (*P* < 0.05).

**Figure 8:** Incidence of adverse vascular events in two groups of patients. ∗ indicates significant difference in diagnostic accuracy versus conventional multimodal MRI images (*P* < 0.05); # means significant difference versus CNN algorithm (*P* < 0.05).

**Figure 9:** Comparison of imaging diagnostic accuracy of different algorithms. ∗ indicates obvious difference compared with the diagnostic accuracy of CTA image before segmentation algorithm processing (*P* < 0.05).

## Data Availability

The data used to support the findings of this study are available from the corresponding author upon request.

## References

[1] Khamis R. Y., Ammari T., Mikhail G. W., Mikhail G. W. (2016). Gender differences in coronary heart disease. *Heart*.

[2] Anderson L., Thompson D. R., Oldridge N. (2016). Exercise-based cardiac rehabilitation for coronary heart disease. *Cochrane Database of Systematic Reviews*.

[3] Perdoncin E., Duvernoy C. (2017). Treatment of coronary artery disease in women. *Methodist DeBakey Cardiovascular Journal*.

[4] Houston M. (2018). The role of noninvasive cardiovascular testing, applied clinical nutrition and nutritional supplements in the prevention and treatment of coronary heart disease. *Therapeutic Advances in Cardiovascular Disease*.

[5] Al-Lamee R. K., Nowbar A. N., Francis D. P. (2019). Percutaneous coronary intervention for stable coronary artery disease. *Heart*.

[6] Doenst T., Haverich A., Serruys P. (2019). PCI and CABG for treating stable coronary artery disease: JACC review topic of the week. *Journal of the American College of Cardiology*.

[7] Santin A. D., Deng W., Frumovitz M. (2020). Phase II evaluation of nivolumab in the treatment of persistent or recurrent cervical cancer (NCT02257528/NRG-GY002). *Gynecologic Oncology*.

[8] Burzotta F., Lassen J. F., Banning A. P. (2018). Percutaneous coronary intervention in left main coronary artery disease: the 13th consensus document from the European Bifurcation Club. *EuroIntervention*.

[9] Nelson C. P., Goel A., Butterworth A. S. (2017). Association analyses based on false discovery rate implicate new loci for coronary artery disease. *Nature Genetics*.

[10] Kolkailah A. A., Alreshq R. S., Muhammed A. M., Zahran M. E., Anas El-Wegoud M., Nabhan A. F. (2018). Transradial versus transfemoral approach for diagnostic coronary angiography and percutaneous coronary intervention in people with coronary artery disease. *Cochrane Database of Systematic Reviews*.

[11] Collet V., Onuma Y., Andreini D. (2018). Coronary computed tomography angiography for heart team decision-making in multivessel coronary artery disease. *Eur Heart J.*.

[12] Chang H. J., Lin F. Y., Lee S. E. (2018). Coronary atherosclerotic precursors of acute coronary syndromes. *Journal of the American College of Cardiology*.

[13] Nørgaard B. L., Leipsic J., Gaur S. (2014). Diagnostic performance of noninvasive fractional flow reserve derived from coronary computed tomography angiography in suspected coronary artery disease: the NXT trial (Analysis of Coronary Blood Flow Using CT Angiography: Next Steps). *Journal of the American College of Cardiology*.

[14] Le Q. C., Arimura H., Ninomiya K., Kabata Y. (2020). Radiomic features based on Hessian index for prediction of prognosis in head-and-neck cancer patients. *Scientific Reports*.

[15] Qiu S., Lian J., Ding Y., Zhou T., Liang T. (2021). Algorithm of pulmonary vascular segment and centerline extraction. *Computational and Mathematical Methods in Medicine*.

[16] Wang C., Oda M., Hayashi Y. (2020). Tensor-cut: a tensor-based graph-cut blood vessel segmentation method and its application to renal artery segmentation. *Medical Image Analysis*.

[17] Hokkinen L., Mäkelä T., Savolainen S., Kangasniemi M. (2021). Evaluation of a CTA-based convolutional neural network for infarct volume prediction in anterior cerebral circulation ischaemic stroke. *European Radiology Experimental*.

[18] Chen Y., Fan S., Chen Y. (2021). Vessel segmentation from volumetric images: a multi-scale double-pathway network with class-balanced loss at the voxel level. *Medical Physics*.

[19] Pereira S., Pinto A., Alves V., Silva C. A. (2016). Brain tumor segmentation using convolutional neural networks in MRI images. *IEEE Transactions on Medical Imaging*.

[20] Giannini F., Candilio L., Mitomo S. (2018). A practical approach to the management of complications during percutaneous coronary intervention. *JACC: Cardiovascular Interventions*.

[21] Ahmad Y., Howard J. P., Arnold A. (2020). Complete revascularization by percutaneous coronary intervention for patients with ST-segment-elevation myocardial infarction and multivessel coronary artery disease: an updated meta-analysis of randomized trials. *Journal of the American Heart Association*.

[22] Al'Aref S. J., Singh G., Choi J. W. (2020). A boosted ensemble algorithm for determination of plaque stability in high-risk patients on coronary CTA. *JACC Cardiovascular Imaging*.

[23] Watts G. F., Sullivan D. R., Hare D. L. (2021). Integrated guidance for enhancing the care of familial hypercholesterolaemia in Australia. *Heart, Lung and Circulation*.

